The article "lncRNA MSC-AS1 Aggravates Diabetic Nephropathy by Regulating the miR-325/CCNG1 Axis" was retracted in 2023. Reasons: signs of a paper mill; suspected computer-generated content; unreliable results or conclusions; concerns about the data.

# lncRNA MSC-AS1 Aggravates Diabetic Nephropathy by Regulating the miR-325/CCNG1 Axis

**DOI:** 10.1155/2022/2279072

**Published:** 2022-01-25

**Authors:** Hongtu Zhao, Yuanyuan Cui, Fuqing Dong, Wencong Li

**Affiliations:** ^1^Department of Endocrinology, 960th Hospital Chinese Peoples Liberat Army, Tai'an, Shandong, China; ^2^Department of Endocrine Rheumatology and Immunology, People's Hospital of Gaotang County, Liaocheng, Shandong, China; ^3^Department of Endocrinology, Zibo Zhoucun People's Hospital, Zibo, Shandong, China; ^4^Department of Endocrinology, Shandong Provincial Third Hospital, Jinan, Shandong, China

## Abstract

**Background:**

Diabetic nephropathy (DN) is the most common microvascular complication of diabetes and has become the second leading cause of end-stage renal disease in the world. This study aims to clarify the regulatory mechanism of the lncRNA MSC-AS1/miR-325/cyclin G1 (CCNG1) axis in DN.

**Methods:**

The regulatory mechanism of lncRNA MSC-AS1/miR-325/CCNG1 was evaluated by RT-qPCR, CCK-8 assay, flow cytometry assay, RNA pull-down assay, ELISA, and western blot assay.

**Results:**

Upregulation of lncRNA MSC-AS1 was detected in DN patients and HRMC cells treated with high glucose (HG). Knockdown of lncRNA MSC-AS1 reduced the proliferation, fibrosis, and inflammation of HRMC cells induced by HG. In addition, lncRNA MSC-AS1 acts as a miR-325 sponge in the DN. CCNG1 is the direct target of miR-325, which can be positively regulated by lncRNA MSC-AS1 in DN. More importantly, downregulation of miR-325 and upregulation of CCNG1 can attenuate the protective effect of lncRNA MSC-AS1 knockdown on DN.

**Conclusion:**

lncRNA MSC-AS1 aggravates DN by downregulating miR-325 and upregulating CCNG1.

## 1. Introduction

Diabetic nephropathy (DN) is a kidney disease caused by diabetes and is the most common microvascular complication of diabetes [1]. DN has become the second leading cause of end-stage renal disease in the world and is prone to major vascular events [2]. DN can cause proteinuria, edema, and hypertension. In severe cases, it can lead to kidney failure and life-threatening [3]. The occurrence of DN is related to metabolic status, oxidative stress, immune inflammatory factors, genetic factors, and changes in renal hemodynamics [4]. Controlling these pathogenic factors is an important way to prevent the occurrence of DN. Therefore, exploring the mechanisms affecting these pathogenic factors is beneficial to patients with DN.

Recently, more and more studies have shown that long noncoding RNA (lncRNA) is involved in the pathogenesis of human diseases including DN. Qin et al. reported that lncRNA PVT1 regulated HG-induced viability, oxidative stress, fibrosis, and inflammation in DN through the miR-325-3p/Snail1 axis [5]. It has been found that knockdown of lncRNA NORAD inhibits the proliferation, inflammation, and fibrosis of human mesangial cells under HG conditions by regulating the miR-485/NRF1 axis [6]. lncRNA HCP5 knockdown has been found to inhibit HG-induced excessive proliferation, fibrosis, and inflammation of human glomerular mesangial cells by regulating the miR-93-5p/HMGA2 axis [7]. lncRNA MSC-AS1 has also been reported to regulate the occurrence of various human diseases. For example, lncRNA MSC-AS1 upregulates BMP2 through spongy microRNA-140-5p to promote osteogenic differentiation and reduce osteoporosis [8]. lncRNA MSC-AS1 activated the Wnt/*β*-catenin signaling pathway and regulated cell proliferation and migration in renal clear cell carcinoma through miR-3924/WNT5A [9]. However, the function of lncRNA MSC-AS1 in DN is still unclear and needs further exploration.

Here, miR-325 is predicted to be the downstream target of lncRNA MSC-AS1. MiR-325 has been found to regulate HG-induced viability, oxidative stress, fibrosis, and inflammation in DN through the mediation of lncRNA PVT1 [5]. In addition, lncRNA MSC-AS1 promoted the progression of colorectal cancer by regulating the miR-325/TRIM14 axis [10]. However, the interaction of lncRNA MSC-AS1 and miR-325 in DN has not been reported in previous studies. Therefore, this study aims to explain the regulatory mechanism of lncRNA MSC-AS1/miR-325 in DN. In addition, this study also investigated the relationship between cyclin G1 (CCNG1) and lncRNA MSC-AS1. CCNG1 has been reported to participate in the pathogenesis of human diseases by mediating lncRNA or miRNA. For example, lncRNA OIP5-AS1 promoted the progression of ovarian cancer by regulating CCNG1 [11]. MiR-122-5p inhibited cell proliferation, migration, and invasion by targeting CCNG1 in pancreatic ductal adenocarcinoma [12]. Moreover, silencing CCNG1 has been found to protect MPC-5 cells from HG-induced proliferation inhibition and apoptosis promotion through the MDM2/*p*53 signaling pathway [13]. However, the regulatory mechanism of lncRNA MSC-AS1/miR-325/CCNG1 in DN is still unknown.

Therefore, this study aims to clarify the regulatory role of lncRNA MSC-AS1/miR-325/CCNG1 axis in DN. At the same time, the effects of lncRNA MSC-AS1 on the proliferation, fibrosis, and inflammation of HRMC cells induced by HG were investigated. This study may help us better understand the pathogenesis of DN.

## 2. Materials and Methods

### 2.1. Serum Samples

30 DN patients and 30 normal subjects in Shandong Provincial Third Hospital were involved in this study. All participants provided written informed consent. This study was approved by the Ethics Committee of Shandong Provincial Third Hospital (Hum2019-06). The clinical characteristics of DN patients and normal people are shown in Table 1. The blood samples collected from these DN patients and normal people were centrifuged to obtain serum samples. Serum samples are stored in a refrigerator at − 80°C until used.

### 2.2. Inclusion and Exclusion Criteria

Inclusion criteria are as follows: (1) age ≥50 years; (2) all meet the relevant diagnostic criteria for DN set by the WHO; (3) DN stage is stage III or IV; and (4) 24 h urinary albumin excretion rate (urinary albumin excretion rates, UAER) is 20–200 *μ*g/min.

Exclusion criteria are as follows: (1) various types of edemas that are difficult to treat; (2) serum alanine aminotransferase (GPT) level is more than twice the normal level; (3) patients with myocardial infarction, infection, or nephritis that cause elevated levels of urine microalbumin; (4) patients with malignant tumors; and (5) women in pregnancy or lactation.

### 2.3. DN Cell Model

Human renal mesangial cell line HRMC (Procell, Wuhan, China) was cultured in a matched dedicated complete medium (CM-H067; Procell) at 37°C with 5% CO_2_. Next, HRMC cells were cultured in HG medium (30 mM D-glucose) to prepare a DN cell model. HRMC cells cultured in normal glucose medium (NG, 5.5 mM D-glucose) were used as a control.

### 2.4. Cell Transfection

mscMSCAS1 siRNA or overexpression vector, miR-325 mimics or inhibitors, and CCNG1 siRNA were purchased from RiboBio (Guangzhou, China). HRMC cells were transfected with the aforementioned agents using Lipofectamine 2000 at 37°C for 48 h.

### 2.5. RT-qPCR

TRIzol reagent (Invitrogen, Carlsbad, CA, USA) was used to extract total RNA from serum or HRMC cells. The synthesis of cDNA was performed using the miRNA Reverse Transcription kit (Invitrogen). Next, qPCR analysis was performed with the Applied Biosystems SYBR™ Green PCR Master Mix (Invitrogen). U6 or GAPDH is used as an internal reference standard. The 2^−ΔΔCt^ method was used to analyze the expression of MSC-AS1, miR-325, and CCNG1. The sequences of the primers used are as follows: MSC-AS1 forward, 5′-GAC TCT CCT ACT GGT GCT TGG T-3′ and reverse, 5′-CAC TGC CTG GTG AGC CTG TT-3′; miR-325 forward, 5′-CGC AAA GTG CTG TTC GTG C-3′ and reverse, 5′-AGT GCA GGG TCC GAG GTA TT-3′; CCNG1 forward, 5′-TTC AGC CCA GGG ACA ACC T-3′ and reverse, 5′-TCT TGT TTT TGC TGC CTT TGG-3′; U6 forward: 5′-CGC TTC GGC AGC ACA TAT AC-3′, reverse: 5′-TTC ACG AAT TTG CGT GTC AT-3′; and GAPDH forward, 5′-GGT GAA GGT CGG AGT CAA CG-3′, and reverse: 5′-CAA AGT TGT CAT GGA TGH ACC-3′.

### 2.6. CCK-8 Assay

Cell viability was detected by the CCK-8 assay. The treated HRMC cells (2000 cells/well) were cultured in 96-well plates for 24, 48, and 72 h, respectively. Afterwards, the cells were treated with 10 *μ*L of CCK-8 reagent (Dojindo, Kumamoto, Japan) for 2 h. A microplate reader (Bio-Rad, Hercules, CA, USA) was used to estimate the optical density at 450 nm.

### 2.7. Flow Cytometry Assay

The treated HRMC cells were harvested and washed with phosphate buffered saline (PBS). Then, the cells were incubated with Annexin V-FIFC binding buffer (Beyotime, Shanghai, China) and propidium iodide (PI, Beyotime) according to the protocol. A flow cytometer (Beckman, Miami, CA, USA) was used to detect the rate of apoptosis.

### 2.8. RNA Pull-Down Assay

First, Bio-miR-325 or Bio-NC (RiboBio) was transfected into HRMC cells for 48 h. Then, the transfected cells were treated with the lysis buffer from the Pierce™ Magnetic RNA-Protein Pull-Down Kit (Thermo Fisher Scientific). Finally, the enrichment of MSC-AS1 or CCNG1 in the pull-down compounds was measured by qRT-PCR.

### 2.9. Western Blot Assay

RIPA lysis buffer (Thermo Fisher Scientific) was used to extract total protein. The protein was separated by 10% SDS-PAGE and then transferred to a PVDF membrane. Next, the separated proteins were blocked with 5% skim milk and incubated overnight with primary antibodies of FN (Abcam, ab2413), Col IV (Abcam, ab86042), Col I (Abcam, ab138492), and GAPDH (Abcam, AB9485). Afterwards, the Goat Anti-rabbit IgG H&L (HRP) secondary antibody (Abcam, ab205718) continued to incubate the protein. Protein blots were detected by an enhanced chemiluminescence kit (Beyotime).

### 2.10. ELISA

TNF-*α*, IL-6, and IL-1*β* levels were assessed by using the Human TNF-*α* ELISA Kit (Abcam), Human IL-6 ELISA Kit (Abcam), and Human IL-1*β* ELISA Kit (Abcam). The experimental procedure is performed according to the protocols.

### 2.11. Statistical Analysis

All experiments were repeated three times. Statistical analysis was performed using GraphPad Prism 6.0 and SPSS 20.0. The data are shown as mean ± SD. The differences between groups were analyzed by Student's *t*-test or one-way ANOVA, followed by Tukey's post hoc test. *P* < 0.05 indicates statistical significance.

## 3. Results

### 3.1. lncRNA MSC-AS1 Knockdown Alleviates HG-Induced Proliferation, Fibrosis, and Inflammation of HRMC Cells

The expression of lncRNA MSC-AS1 was detected in DN serum samples and DN cell models. We found that the expression of lncRNA MSC-AS1 was higher than that of normal subjects (*P* < 0.05) (Figure 1(a)). Compared with NG-treated HRMC cells, lncRNA MSC-AS1 was upregulated in HG-treated HRMC cells (*P* < 0.01) (Figure 1(b)). To explore the potential role of MSC-AS1 in DN, si-MSC-AS1 was transfected into HG-treated HRMC cells. RT-qPCR showed that the expression of MSC-AS1 was significantly reduced (*P* < 0.01) (Figure 1(c)), indicating that si-MSC-AS1 is effective. Functionally, the CCK-8 assay showed that compared with NG, HG significantly promoted the proliferation of HRMC cells, while si-MSC-AS1 inhibited HG-induced proliferation (*P* < 0.01) (Figure 1(d)). At the same time, the apoptotic rate of HRMC cells was inhibited by HG but was enhanced by MSC-AS1 knockdown (*P* < 0.01) (Figure 1(e)). In addition, we found that the protein expression of cell fibrosis-related markers (FN, Col IV, and Col I) was increased in HG-treated HRMC cells, but was inhibited by si-MSC-AS1 (*P* < 0.01) (Figure 1(f)). In addition, we found that TNF-*α*, IL-6, and IL-1*β* levels were enhanced by HG but suppressed by MSC-AS1 knockdown (*P* < 0.01) (Figure 1(g)). Collectively, downregulation of lncRNA MSC-AS1 can alleviate the proliferation, fibrosis, and inflammation of HRMC cells induced by HG.

### 3.2. lncRNA MSC-AS1 Functions as a miR-325 Sponge

StarBase (http://starbase.sysu.edu.cn/, Figure 2(a)) predicts that miR-325 is the target of lncRNA MSC-AS1. Then, an RNA pull-down assay was performed to verify the relationship between MSC-AS1 and miR-325. We found that BiomiR-325 can pull a high abundance of MSC-AS1 down in HRMC cells (*P* < 0.01) (Figure 2(b)). In HG-treated HRMC cells, miR-325 expression was reduced by the MSC-AS1 vector and increased by si-MSC-AS1 (*P* < 0.01) (Figure 2(c)). At the same time, miR-325 overexpression inhibited MSC-AS1 expression, while miR-325 downregulation promoted MSC-AS1 expression in HG-treated HRMC cells (*P* < 0.01) (Figure 2(d)). In addition, miR-325 expression was detected in DN serum samples. Downregulation of miR-325 was detected (*P* < 0.01) (Figure 2(e)) and was negatively correlated with the expression of MSC-AS1 in DN serum samples (*P* < 0.01) (Figure 2(f)). Taken together, the lncRNA MSC-AS1 acts as a miR-325 sponge in DN.

### 3.3. CCNG1 Is a Direct Target of miR-325

The TargetScan database (http://www.targetscan.org) shows that CCNG1 has a binding site for miR-325 (Figure 3(a)). In addition, compared with Bio-NC, Bio-miR-325 can enrich a high abundance of CCNG1 (*P* < 0.01) (Figure 3(b)). Moreover, CCNG1 expression was inhibited by miR-325 overexpression and promoted by miR-325 downregulation in HG-treated HRMC cells (*P* < 0.01) (Figure 3(c)). These results indicate that miR-325 can bind to CCNG1 in HG-treated HRMC cells. In addition, CCNG1 expression was increased in DN serum samples compared with normal subjects (*P* < 0.01) (Figure 3(d)). And CCNG1 expression was negatively correlated with miR-325 expression but positively correlated with lncRNA MSC-AS1 expression in DN serum samples (*P* < 0.01) (Figures 3(e) and 3(f)). At the same time, CCNG1 expression was inhibited by si-MSC-AS1 and promoted by MSC-AS1 vector in HG-treated HRMC cells (*P* < 0.01) (Figure 3(g)). In short, CCNG1 is the direct target of miR-325 and can be positively regulated by the lncRNA MSC-AS1 in DN.

### 3.4. lncRNA MSC-AS1 Aggravates DN by Downregulating miR-325 and Upregulating CCNG1

In order to investigate the interaction between lncRNA MSC-AS1 and miR-325 or CCNG1, the CCNG1 vector or miR-325 inhibitor was transfected into HG-treated HRMC cells with si-MSC-AS1. RT-qPCR showed that the CCNG1 vector or miR-325 inhibitor restored the decreased expression of MSC-AS1 induced by its siRNA (Figure 4(a). In HG-treated HRMC cells, miR-325 downregulation or CCNG1 upregulation restored cell proliferation inhibited by si-MSC-AS1 (Figure 4(b)). And si-MSC-AS1-stimulated apoptosis was inhibited by downregulation of miR-325 or upregulation of CCNG1 in HG-treated HRMC cells (Figure 4(c)). Compared with HG-treated HRMC cells containing si-MSC-AS1, the protein levels of FN, Col IV, and Col I were largely recovered in HG-treated HRMC cells with si-MSC-AS1+CCNG1 vector or si-MSC-AS1+miR-325 inhibitor (Figure 4(d)). Furthermore, MSC-AS1 knockdown prevented the release of TNF-*α*, IL-6, and IL-1*β*, while miR-325 downregulation or CCNG1 upregulation restored the release of these proinflammatory factors (Figure 4(e)). These results indicate that lncRNA MSC-AS1 aggravates DN through downregulation of miR-325 and upregulation of CCNG1.

## 4. Discussion

In this study, we found that lncRNA MSC-AS1 expression was significantly upregulated in DN serum samples and HG-treated HRMC cells. Functionally, knockdown of lncRNA MSC-AS1 alleviated HG-induced proliferation, fibrosis, and inflammation of HRMC cells. In terms of mechanism, it was found that lncRNA MSC-AS1 competitively binds to miR-325, which in turn upregulates the expression of CCNG1. More importantly, rescue experiments showed that lncRNA MSC-AS1 aggravated DN by downregulating miR-325 and upregulating CCNG1. All these results indicate that the lncRNA MSC-AS1 is a risk factor for patients with DN.

A large number of studies have shown that lncRNA MSC-AS1 promoted the malignant behavior of human cancers, such as proliferation, apoptosis, migration, and invasion [14–16]. These findings indicate that the lncRNA MSC-AS1 plays a vital role in the occurrence and development of cancer. Besides, it has been reported that lncRNA MSC-AS1 promoted cell proliferation and migration in renal clear cell carcinoma through miR-3924/WNT5A [9]. Wan et al. found that lncRNA MSC-AS1 may play an important role in the development of diabetic vasculopathy (DV) and is expected to become a therapeutic target for DV [17]. These studies indicate that the lncRNA MSC-AS1 may be involved in diabetic and kidney-associated diseases. Consistently, our study proposed for the first time that lncRNA MSC-AS1 expression was increased in DN serum samples and HG-treated HRMC cells. Knockdown of lncRNA MSC-AS1 inhibited HG-induced proliferation, fibrosis, and inflammation of HRMC cells. These results indicate that the lncRNA MSC-AS1 is a potential pathogenic factor for DN.

In terms of mechanism, it is found that lncRNA MSC-AS1 has a miR-325 binding site. And lncRNA MSC-AS1 acts as a miR-325 sponge in DN. Consistent with our results, lncRNA MSC-AS1 has been proposed to promote the progression of colorectal cancer through sponging miR-325 [10]. In addition, downregulation of miR-325 was found in DN serum samples. And downregulation of miR-325 weakened the protective effect of lncRNA MSC-AS1 knockdown on DN, indicating that overexpression of miR-325 can block the development of DN. Similar to our results, miR-325-3p has been reported to inhibit renal inflammation and fibrosis by targeting CCL19 in DN [18]. These findings indicate that overexpression of miR-325 is beneficial to control DN. Furthermore, CCNG1 was found to be a direct target of miR-325. And miR-325 inhibited CCNG1 expression by binding to its 3′UTR. Our data also showed that CCNG1 expression was significantly upregulated in DN serum samples. Functionally, CCNG1 overexpression restored lncRNA MSC-AS1 knockdown-inhibited HRMC cell proliferation, fibrosis, and inflammation. Consistent with our results, Chen et al. reported that downregulation of CCNG1 had a protective effect on DN, and its mechanism was related to the MDM2-p53 pathway [13]. All these findings emphasize that CCNG1 is the pathogenic factor of DN.

## 5. Conclusion

To conclude, lncRNA MSC-AS1 promotes HG-mediated DN progression in mesangial cells by regulating the miR-325/CCNG1 axis. This study may help us better understand the pathogenesis of DN. However, our conclusion has not been confirmed *in vivo*. Therefore, we will design *in vivo* experiments in the future to further verify our conclusions.

## Figures and Tables

**Figure 1:** LncRNA MSC-AS1 knockdown alleviates HG-induced proliferation, fibrosis, and inflammation of HRMC cells. (a) The expression of MSC-AS1 in serum samples from DN patients and normal subjects (*n* = 30). (b) The expression of MSC-AS1 in HG- and NG-treated HRMC cells. (c) The expression of MSC-AS1 in HG-treated HRMC cells with its siRNA. (d, e) Cell proliferation and apoptosis were detected in the NG, HG, and HG + si-MSC-AS1 groups. (f) Cell fibrosis was assessed by the levels of FN, Col IV, and Col I in the NG, HG, and HG + si-MSC-AS1 groups. (g) The release of TNF-*α*, IL-6, and IL-1*β* was examined in the NG, HG, and HG + si-MSC-AS1 groups. ^*∗*^*P* < 0.05^*∗∗*^*P* < 0.01.

**Figure 2:** lncRNA MSC-AS1 functions as a miR-325 sponge. (a) The binding sites between MSC-AS1 and miR-325. (b) The relationship between MSC-AS1 and miR-325 was verified by pull-down assay. (c) MiR-325 expression was detected in HG-treated HRMC cells with MSC-AS1 siRNA and vector. (d) MSC-AS1 expression was measured in HG-treated HRMC cells containing miR-325 mimics or inhibitors. (e) MiR-325 expression was detected in DN patients and normal subjects (*n* = 30). (f) A negative correlation between MSC-AS1 and miR-325 expression was found in DN patients (*n* = 30). ^*∗*^*P* < 0.05, ^*∗∗*^*P* < 0.01.

**Figure 3:** CCNG1 is a direct target of miR-325. (a) The binding sites between miR-325 and CCNG1. (b) The relationship between miR-325 and CCNG1 was confirmed by pull-down assay. (c) CCNG1 expression was measured in HG-treated HRMC cells containing miR-325 mimics or inhibitors. (d) CCNG1 expression was detected in DN patients and normal subjects. (e) A negative correlation between CCNG1 and miR-325 expression was identified in DN patients (*n* = 30). (f) A positive correlation between MSC-AS1 and CCNG1 expression was detected in DN patients (*n* = 30). (g) CCNG1 expression was assessed in HG-treated HRMC cells with MSC-AS1 siRNA and vector. ^*∗*^*P* < 0.05, ^*∗∗*^*P* < 0.01.

**Figure 4:** lncRNA MSC-AS1 aggravates DN by downregulating miR-325 and upregulating CCNG1. (a) The expression of MSC-AS1 was detected in HG, HG + si-MSC-AS1, HG + si-MSC-AS1+miR-325 inhibitor, and HG + si-MSC-AS1+CCNG1 vector groups. (b, c) Cell proliferation and apoptosis were detected in HG, HG + si-MSC-AS1, HG + si-MSC-AS1+miR-325 inhibitor, and HG + si-MSC-AS1+CCNG1 vector groups. (d) The levels of FN, Col IV, and Col I were measured in HG, HG + si-MSC-AS1, HG + si-MSC-AS1+miR-325 inhibitor, and HG + si-MSC-AS1+CCNG1 vector groups. (e) TNF-*α*, IL-6, and IL-1*β* levels were examined in HG, HG + si-MSC-AS1, HG + si-MSC-AS1+miR-325 inhibitor, and HG + si-MSC-AS1+CCNG1 vector groups. ^*∗*^*P* < 0.05, ^*∗∗*^*P* < 0.01.

**Table 1:** Clinical characteristics of patients with DN and healthy controls.

Characteristics	Normal	DN
Male	16	17
Female	14	13
Age (y)	51.6 ± 5.8	50.4 ± 4.8
BMI (kg/m2)	21.9 ± 3.1	24.5 ± 3.5
SBP (mm hg)	110.6 ± 14.8	157.8 ± 26.4^*∗*^
DBP (mm hg)	81.2 ± 6.3	85.6 ± 10.8^*∗*^
FPG (mM)	4.8 ± 2.1	8.4 ± 2.0^*∗*^
HbA1c (%)	5.3 ± 1.6	8.6 ± 2.2^*∗*^
TC (mM)	5.01 ± 1.2	6.27 ± 1.6^*∗*^
TG (mM)	1.28 ± 1.0	2.42 ± 1.1^*∗*^
LDL-C (mM)	3.05 ± 1.12	3.68 ± 1.16^*∗*^
BUN (mM)	5.20 ± 1.29	8.25 ± 1.44^*∗*^
SCr (*μ*M)	60.16 ± 11.23	122.2 ± 20.4^*∗*^

^*∗*^ *P* < 0.05.

## Data Availability

Data to support the findings of this study are available on reasonable request from the corresponding author.
